# Efficacy Analysis of Team-Based Nursing Compliance in Young and Middle-Aged Diabetes Mellitus Patients Based on Random Forest Algorithm and Logistic Regression

**DOI:** 10.1155/2022/3882425

**Published:** 2022-07-29

**Authors:** Dongni Qian, Hong Gao

**Affiliations:** ^1^Department of Endocrinology, The Third People's Hospital of Hefei, Hefei 230022, China; ^2^Nursing Department, The Third People's Hospital of Hefei, Hefei 230022, China

## Abstract

**Objective:**

Long-term hyperglycemia in young and middle-aged diabetic patients can be complicated with diabetic ketoacidosis, stroke, myocardial infarction, infection, and other complications. The objective was to explore the application value of machine learning in predicting the recurrence risk of young and middle-aged diabetes patients with team-based nursing intervention.

**Methods:**

Clinical data of 80 patients with diabetes treated in the Department of Endocrinology from 2019 to 2020 were retrospectively collected. The data set was divided into 70% training set (*n* =56) and 30% test set (*n* =24). All the selected research cases were intervened by the team-based management mode involving family and clinical doctors and nurses. The degree of diabetes knowledge learning, the level of blood glucose changes, and the psychological state of the patients were evaluated. The random forest (RF) algorithm and logistic regression prediction model were constructed to predict the risk factors of diabetes recurrence.

**Results:**

There was no significant difference in the degree of diabetes knowledge learning, the level of blood glucose changes, and the psychological state between the training set and the test set (*P* > 0.05). The FPG, HbA1c, and 2hPG of recurrence group patients were significantly higher than those of nonrecurrence group patients, and the difference was statistically significant (*P* < 0.05). In descending order of importance based on the RF algorithm prediction model were glucose, BMI, age, insulin, pedigree function, skin thickness, and blood diastolic pressure. The accuracy of RF and logistic regression prediction models is 81.46% and 80.21%, respectively.

**Conclusion:**

The team-based nursing model has a good effect on the blood glucose control level of middle-aged and young diabetic patients. Age, BMI, and glucose values are risk factors for diabetes. The SF algorithm has a good effect on predicting the risk of diabetes, which is worthy of further clinical application.

## 1. Introduction

Young and middle-aged diabetes mellitus is a group of metabolic diseases characterized by chronic hyperglycemia caused by insulin secretion or utilization disorder caused by multiple causes [1]. Long-term hyperglycemia significantly increases and accelerates the risk of complications such as diabetic ketoacidosis, stroke, myocardial infarction, and infection [2], which seriously affects the life and quality of life of patients, and even endangers their lives [3]. According to relevant research and analysis, effective blood sugar control can reduce the related end-point events of diabetic patients, including the risk of microvascular complications decreased by 25%, and the risk of myocardial infarction and sudden death decreased by 16% [4]. Therefore, blood glucose control is of great clinical significance for the prevention of various complications.

With the improvement of living standard and the change of lifestyle, the incidence of diabetes is increasing, and it is becoming younger and younger [5, 6]. The number of diabetic patients in China has leapt to the first place in the world. It is estimated that there are about 113.9 million diabetics and 493.4 million people with pre-diabetes among adults aged 18 and above in China [7]. Because the treatment of diabetes is lifelong, the effect of treatment depends to a large extent on whether the patients actively cooperate and master the relevant knowledge and skills. However, this group of people is mostly in the study or work stage, with irregular life, insufficient knowledge, and limited self-care time. After discharge, they often lack continuous care, which leads to poor blood sugar control and even readmission [8, 9].

At present, the international guidelines for the treatment of diabetes all emphasize the principle of comprehensive treatment of diabetes and believe that it is difficult to achieve the long-term and effective control of blood sugar by drug treatment alone [10]. We must take diet, exercise, psychology, need patients to master certain knowledge about diabetes, and actively participate in active cooperation with treatment, so as to comprehensively and effectively control diabetes [11]. Studies have shown that the team-based management intervention of young and middle-aged diabetic families with poor compliance can significantly improve the patients' condition [12]. To our knowledge, there is still little research on how to do an excellent job in team-based family and clinical care management. The team-based nursing mode is a team-based management care approach that includes family clinicians and nurses. Therefore, based on machine learning, this study discusses the relevance of team-based nursing mode to the rate of reaching the standard of blood glucose control and knowledge awareness of young and middle-aged diabetes patients. In addition, we also discussed the adverse factors affecting the recurrence of blood glucose, to provide reference for the prevention and treatment of diabetes.

## 2. Materials and Methods

### 2.1. Research Object

A total of 80 young and middle-aged diabetes patients admitted to the Department of Endocrinology of our hospital from September 2019 to December 2020 were selected as the research object. Inclusion criteria: (1) Diabetes was confirmed by OGTT or steamed bread meal test, including type 1 diabetes, type 2 diabetes, gestational diabetes, and other special types of diabetes. (2) Hospitalized patients in the Endocrinology Department. (3) Patients who had a fixed address within 1 year after discharge and had communication tools to cooperate with the implementation of management nursing can establish a complete follow-up record. Exclusion criteria: (1) Patients who refused to monitor blood glucose after discharge. (2) Patients who refused to return visit on time. (3) Complicated with other serious end-stage diseases. (4) Cognitive and language dysfunction. The study plan was submitted to the hospital ethics committee for approval, and all patients signed informed consent.

### 2.2. Research Method

All the selected research cases were intervened by the team-based management mode involving family, clinical doctors, and nurses, and follow-up guidance was given according to time nodes. The team-based management nursing method involves family clinical doctors and nurses, establishing individual follow-up files, urging patients to regularly monitor blood glucose, blood lipid, blood pressure, glycation, etc. According to the targeted intensive rehabilitation guidance of the follow-up time nodes, and consulting doctors in real time to properly adjust the dosage and types of drugs according to patients' personal conditions, through tracking and interfering with patients' out-of-hospital compliance behavior, urging patients to know the knowledge related to diabetes health education, guiding the establishment of a scientific lifestyle, and guiding patients to adjust the effect of drug taking individually.

The baseline data of patients were collected through the hospital information system, including gender, age, body mass index (BMI), marital status, insulin level, blood glucose, pediatrician function, skin thickness, blood diabetic pressure, and pulse. Through telephone follow-up, outpatient follow-up, and out-of-hospital management system follow-up, the patient's blood sugar status was recorded, and the follow-up time was 1 year. Telephone follow-up was conducted by myself and the specialist nurse in the Endocrine and Metabolic Department. Outpatient follow-up was conducted by the outpatient nurses in the Department of Endocrinology and Metabolism. Follow-up of the out-of-hospital management system was carried out by education nurses in the Endocrine Metabolism Department. During the follow-up, data collection, nursing guidance, evaluation, and statistical analysis were conducted.

### 2.3. Evaluation Index

Self-made diabetes health knowledge questionnaire was used to investigate patients' knowledge of diabetes. It is divided into basic knowledge, self-care knowledge, and medical knowledge. There are 4 questions in each aspect, with a score of 1-5. The higher the score, the better the patient's knowledge of diabetes. Then, the changes of blood glucose were detected, including fasting plasma glucose (FPG), glycated hemoglobin A1c (HbA1c), and 2 h postprandial glucose (2hPG). In addition, we also analyzed patients' degree of anxiety and depression. Self-rating anxiety scale (SAS) and self-rating depression scale (SDS) were used to evaluate the psychological state of patients. SAS scores 50 points, with scores of 50~59 points as mild anxiety, 60~69 points as moderate anxiety, and scores over 69 points as severe anxiety. The demarcation value of SDS is 53 points, with a score of 53~62 points being mild depression, a score of 63~72 points being moderate depression, and a score of more than 73 points being severe depression.

### 2.4. Establishment of Prediction Model

In this study, the data set was divided into 70% training set (*n* =56) and 30% test set (*n* =24). The optimal parameters of the model were obtained by 5-fold crossover validation. The test set data evaluates the training set data to evaluate the prediction efficiency of the model. Then, according to the recurrence of patients, the training set was divided into recurrence group and nonrecurrence group. There were 21 patients in the recurrent group and 35 patients in the nonrecurrent group. The recurrence rate was 26.3%.

### 2.5. Logistic Regression Prediction Model

Logistic regression model is the most widely used multivariate quantitative analysis method for regression analysis of binary dependent variables, which can have both continuous independent variables and classified independent variables [13]. Through logistic regression analysis, the weight of independent variables can be obtained to predict the possibility of events, and the formula is as follows:

(1) $$\begin{array}{c} P\left(Y_{i}=1\;|\;X_{i}\right)=\frac{e^{\alpha +\sum_{i=1}^{k}\beta_{k}X_{ki}}}{1+e^{\alpha +\sum_{i=1}^{k}\beta_{k}X_{ki}}}. \end{array}$$

*Y* is the dependent variable. *X* = [*X*_1_, *X*_2,⋯,_*X*_*k*_] is a set of dependent variables corresponding to *Y*.

### 2.6. Random Forest Prediction Model

The random forest (RF) algorithm is an integration algorithm with a decision tree as a base classifier and obtains the best result by combining multiple decision trees to vote [14]. RF algorithm has the advantages of high accuracy, difficulty in over-fitting, high dimensional feature processing, and high tolerance to noise and abnormal data [14, 15]. The classification result formula of random forest is as follows:

(2) $$\begin{array}{c} H\left(x\right)=\arg\;\max_{\text{y}}\overset{k}{\underset{i=1}{\sum }}I\left(h_{i}\left(x\right)=Y\right). \end{array}$$

*H*(*x*) is a random forest combination classifier model, *h*_*i*_ is a single decision tree model in bagging, and *Y* is a category label.

*OOB* estimation is usually used to measure the generalization error of random forest algorithms. Therefore, *OOB* estimation can be used as an indicator of algorithm classification performance. The generalization error of the random forest algorithm is defined as:

(3) $$\begin{array}{c} PE=P_{X,Y}\left(mg\left(X,Y\right)<0\right). \end{array}$$

The edge function *mg*(*X*, *Y*) is the difference between the average number of correct classifiers and the average number of wrong classifiers. The more significant *mg*(*X*, *Y*) is, the better the algorithm model is.

(4) $$\begin{array}{c} mg\left(X,Y\right)={av}_{k}I\left(h_{k}\left(X\right)=Y\right)-\max_{j\neq Y}{av}_{k}Ij. \end{array}$$

The RF algorithm uses bootstrap re-sampling technology to repeatedly and randomly extract *N* samples from the original training sample set *n* to generate *k* subtraining sets. Each subtraining set builds a regression tree, and the samples that are not extracted each time are called out-of-bag data. RF regression algorithm flow chart is shown in Figure 1.

### 2.7. Statistical Analysis

The SPSS 23.0 statistical software was used for analysis and processing. The measurement data is indicated by $\bar{x}\pm s$, and the comparison between groups is made by *t*-test. The data counting rate was compared by the *χ*^2^ test. The receiver operator characteristic (ROC) curve is used to analyze the prediction efficiency of the model. *P* < 0.05 is statistically significant.

## 3. Results

### 3.1. Comparison of Evaluation Data between Training Set and Test Set

The follow-up results of the patients in the training group and the test group one year after the team-based nursing intervention showed that there was no significant difference in the scores of basic knowledge, self-care knowledge, and medical knowledge of young and middle-aged diabetes (*P* > 0.05) (Table 1). In addition, there was no significant difference in the ratio of FPG, HbA1c, and 2hPG between the patients in the training set and the test set (*P* > 0.05). The detailed results are shown in Figure 2. The scores of patients' psychological state changes in the two data sets showed that the scores of anxiety and depression were low, and there was no significant difference between the two data sets (*P* > 0.05) (Table 2).

### 3.2. Comparison of Assessment Data between the Recurrence and Nonrecurrence Groups in the Training Set

Among the patients in the training set, patients in the recurrence group (*n* =21) and patients in the nonrecurrence group (*n* =35) had better knowledge of diabetes. In addition, the psychological state scores of the two groups were also good, and there was no significant difference (*P* > 0.05) (Table 3). By analyzing the changes in blood sugar, however, the results showed that the FPG, HbA1c, and 2hPG of recurrence group patients were significantly higher than those of nonrecurrence group patients, and the difference was statistically significant (*P* < 0.05) (Figure 3).

### 3.3. Multivariate Logistic Regression Prediction Results

Multivariate logistic regression analysis was performed on the baseline data of patients with diabetes. *a* =0.05 was used as the inclusion condition. 0.10 was used as the exclusion criterion, and the insignificant variables were eliminated by step-step regression. The assignment results are shown in Table 4. The results showed that age, BMI, blood diastolic pressure, insulin, blood glucose, and skin thickness were the risk factors for diabetes recurrence.

### 3.4. Rank the Importance of Predictive Variables

The importance ranking of variables was obtained by the RF algorithm-based diabetes risk prediction model established by the training set. In descending order of importance are blood glucose, BMI, age, insulin, pedigree function, skin thickness, and blood diastolic pressure (Figure 4).

### 3.5. Comparison of the Effectiveness of Prediction Models

The four prediction models constructed in this paper can effectively predict diabetes mellitus. The accuracy of RF and logistic regression prediction models is 81.46% and 80.21%, respectively. The ROC curve is shown in Figure 5.

## 4. Discussion

Diabetes is one of the most common, rapidly growing, and incurable diseases in the world [16]. In addition to its serious complications, diabetes has been linked to the onset of cancer, cognitive impairment, tuberculosis, and depression [17]. In recent years, large cohort studies in China, the United States, and other countries have found that lifestyle and drug interventions for patients with impaired glucose tolerance and pre-diabetes can delay or even reduce the occurrence of diabetes [18]. The risk of diabetes can be predicted by specific models, and the high risk groups can be found as early as possible, and intervention measures can be implemented to improve the health level of the population.

After team-based nursing model, patients had better understanding of basic knowledge, self-care knowledge, and medical knowledge of diabetes. Patients also scored better on psychological status. In addition, the patient's blood glucose levels were also effectively controlled. These results indicate that team-based nursing model has a good effect on the blood glucose control level of middle-aged and young diabetic patients, which is worthy of promotion of clinical work. The results are similar to previous studies [19].

The number of patients with diabetes and its complications is on the rise [20]. The establishment of a prediction model can help doctors timely diagnose patients' disease and its related indicators, carry out interference, and take corresponding measures. In addition, it can also save medical resources and reduce the pressure on patients and society. As can be seen from the importance of characteristic variables of the RF algorithm model, glucose, BMI, and age are more important. It indicated that people with high blood glucose concentration, obesity, and older age are more likely to suffer from diabetes. Recent studies confirm our conclusions [3, 21]. Casanova et al. established a diabetes risk prediction model using the RF algorithm using 8-year follow-up data of 3 633 African Americans from the Jackson Heart Study. The results showed that glucose, BMI, and age were risk factors for diabetes [3]. The risk of diabetes increases with age and BMI, so people who are older or obese should be vigilant about what they eat. Therefore, in the prevention of diabetes, blood glucose concentration and body mass index should be controlled.

It is a hot topic in the research of diabetes risk prediction in the big data era to establish a simple and accurate diabetes risk prediction model by using a data mining algorithm [22, 23]. In this paper, two kinds of diabetes risk prediction models are constructed based on deep learning, which is an efficient diabetes diagnosis technology emerging in recent years [2, 24–26]. The RF algorithm has high prediction performance, and the influence of abnormal data and noise on the algorithm is very low. The logistic regression model is the most widely used multivariate quantitative analysis method for regression analysis of binary dependent variables, which can have both continuous independent variables and classified independent variables [13].

The focus of diabetes prediction model has gradually shifted from high accuracy to high reliability, so that the prediction method can be applied to different populations. Based on the same data set, different diabetes risk prediction models were constructed, and relevant indicators were included to determine the factors of diabetes occurrence. The results show that the RF algorithm model is significantly higher than the logistic regression prediction model (81.46% and 80.21%, respectively). RF algorithm, as an emerging machine learning algorithm, has robust operation, no requirements on data sets, and no over-fitting. It has been widely used in disease risk assessment [27]. Our results also confirm previous conclusions [28].

There are some limitations to this study. First of all, the patient data included in this study were small and single center. Secondly, insufficient predictive variables included in the prediction model may affect the prediction results.

## 5. Conclusion

In conclusion, the team-based nursing model has a good effect on the blood glucose control level of middle-aged and young diabetic patients, which is worthy of promotion of clinical work. Age, BMI, and glucose values are risk factors for diabetes. The RF algorithm has a good effect on predicting the risk of diabetes, which is worthy of further clinical application.

## Figures and Tables

**Figure 1:** Flow chart of RF regression algorithm prediction model.

**Figure 2:** Comparison of blood glucose changes between the two data sets. There was no significant difference in three blood glucose indicators between the two sets (*P* > 0.05).

**Figure 3:** Comparison of blood glucose changes between the recurrence group and nonrecurrence group. There was significant difference in blood glucose between the two groups (all *P* < 0.001).

**Figure 4:** Analysis result of random forest algorithm for diabetes mellitus risk prediction.

**Figure 5:** ROC curves of prediction models constructed by random forest and logistic regression.

**Table 1:** Comparison of knowledge of diabetes between the two data sets.

Data set	Basic knowledge	Self-care knowledge	Medical knowledge
Training set	16.26 ± 3.10	16.44 ± 2.86	16.60 ± 3.15
Test set	16.48 ± 3.21	16.58 ± 2.94	16.64 ± 3.21
*t*	0.288	0.199	0.052
*P*	0.774	0.843	0.959

**Table 2:** Comparison of mental state between the two data sets.

Data set	*N* (%)	SAS	SDS
Training set	56 (70%)	12.35 ± 1.28	12.32 ± 1.17
Test set	24 (30%)	12.46 ± 1.47	12.60 ± 1.22
*t*	—	0.337	0.969
*P*	—	0.737	0.336

**Table 3:** Comparison of knowledge of diabetes and mental state between recurrence group and nonrecurrence group.

Variables	Recurrence group	Nonrecurrence group	*t*	*P*
Knowledge of diabetes	—	—	—	—
Basic knowledge	13.48 ± 3.48	13.57 ± 3.62	0.091	0.928
Self-care knowledge	13.58 ± 3.14	13.69 ± 3.25	0.124	0.902
Medical knowledge	13.12 ± 3.28	13.49 ± 3.64	0.382	0.704
Mental state	—	—	—	—
SAS	19.42 ± 2.81	19.13 ± 2.53	-0.398	0.692
SDS	19.32 ± 2.52	19.14 ± 2.33	-0.271	0.787

**Table 4:** Assignment table of predictive variables based on logistic regression prediction model.

Variable	Variable name	Variable assignment
*Y*	Recurrence of diabetes	—
*X*_1_	Age	Continuous variable
*X*_2_	BMI	Continuous variable
*X*_3_	Blood diastolic pressure	Continuous variable
*X*_4_	Blood glucose	Continuous variable
*X*_5_	Insulin	Continuous variable
*X*_6_	Skin thickness	Continuous variable

## Data Availability

The data used to support the findings of this study are available from the corresponding author upon request.
